# Factors Influencing Cerebrospinal Fluid Leaking following Pituitary Adenoma Transsphenoidal Surgery: A Meta-Analysis and Comprehensive Review

**DOI:** 10.1155/2022/5213744

**Published:** 2022-08-16

**Authors:** Jiao Zhang, Jingyun Liu, Liyan Huang

**Affiliations:** Operating Room, The First Hospital of China Medical University, Shenyang, Liaoning 110001, China

## Abstract

**Background:**

Surgical resection is the main method to treat pituitary adenoma. Cerebrospinal fluid leakage (CSF Leak) is the main complication after transsphenoidal surgery. The impact of postoperative CSF Leak can be predicted in advance, and preventive measures can be taken in time. Clinically, a variety of factors may affect the occurrence of postoperative CSF Leak. In this study, meta-analysis was used to investigate the risk factors of postoperative CSF Leak as a clinical reference.

**Methods:**

The databases PubMed, Medline, Embrase, Cochrane library, CNKI, and CBM were searched for all studies on the risk factors of postoperative CSF Leak. Studies were screened and finally included. The quality of the included studies was assessed by the Newcastle-Ottawa scale. We used Revman 5.4 software to conduct the pooled effect size of every potential statistically significant factor.

**Results:**

13 articles with a total of 5967 patients with pituitary adenoma and 405 cases of postoperative CSF Leak were finally included, accounting for 6.79%. All of the 13 articles had a quality score > 5, indicating good quality. Meta-analysis showed that patient age (OR = 0.71, 95% CI (0.41, 1.20), *P* = 0.20) was not a factor influencing postoperative CSF Leak, while BMI (MD = 2.26, 95% CI (1.31, 3.20), *P* < 0.00001), tumor size (MD = 1.35, 95% CI (0.22, 2.49), *P* = 0.02), whether a second operation was performed (OR = 2.20, 95% CI (1.45, 3.33), *P* = 0.0002), and intraoperative CSF Leak (OR = 8.88, 95% CI (3.64, 21.69), *P* < 0.00001) were risk factors for postoperative CSF Leak in patients. *Discussion*. BMI, tumor size, reoperation, and intraoperative CSF Leak are the risk factors of postoperative CSF Leak. However, not all the factors were covered in this study, it is still worth continuing to deeply investigate in this topic.

## 1. Introduction

Pituitary adenomas are benign tumors arising from the adenohypophyseal cells of the anterior pituitary gland, located in the saddle region in the middle of the base of the brain, and are characterized by slow growth, small local lesions, and nonmetastasis [1]. According to the size of the tumor, pituitary adenomas can be divided into microadenomas (diameter < 10 mm), macroadenomas (diameter ≥ 10 mm), and giant adenomas (diameter ≥ 40 mm). According to the function of the tumor and the characteristics of hormone secretion, pituitary adenomas can be divided into functional pituitary adenomas and nonfunctional pituitary adenomas [2]. The vast majority of pituitary adenomas are nonfunctional pituitary microadenomas. Patients have no symptoms and signs for their whole life and do not need treatment. Only about 0.1%-0.2% of pituitary adenomas will metastasize into pituitary cancer, which is very rare [2]. Among all intracranial tumors, pituitary adenomas account for about 10%-15% and tend to happen to people aged 30-50, and the incidence is independent of gender [3].

Although most microadenomas are asymptomatic, when pituitary tumors cause pituitary hyperfunction or hypofunction, tumor space occupying effect, and pituitary tumor stroke, they will have a negative impact on the human body [4]. The pituitary gland plays a very important role in maintaining endocrine balance in the human body, functional pituitary adenomas may cause excessive secretion of hormones and cause hyperpituitarism, and the local mass effect of tumors may cause headache, decreased visual acuity, and hydrocephalus symptoms, while giant adenomas may compress intracranial tissues and lead to hypopituitarism [5]. Therefore, when patients have headache, decreased vision, or visual impairment, combined with sexual dysfunction caused by endocrine abnormalities (male), menopause or lactation stop (female), and abnormal obesity, they should seek medical examination in time to diagnose the existence of pituitary adenoma.

Surgical resection is the mainstay of treatment for pituitary adenomas, and endoscopic transsphenoidal surgery (ETS) has been widely used because of its less trauma and good safety, but this procedure also has complications such as bleeding, infection, cerebrospinal fluid leakage (CSF Leak), and decreased visual acuity [6]. Transsphenoidal surgery has been plagued by cerebrospinal fluid leak and intracranial infection since its inception in the 20th century. It was once abandoned because of the high risk of infection, but with the help of antibiotics, the risk of infection has been greatly reduced. With the application of endoscopic technology in surgery, the visual angle and field of vision during surgery are clearer, which makes transsphenoidal surgery popular again and widely used in neurosurgery today [7].

However, the application of new technology cannot completely avoid the occurrence of surgical complications. The common complications of transsphenoidal surgery include cerebrospinal fluid leak, epistaxis, dysosmia, and sinusitis. CSF Leak is the main complication of transsphenoidal surgery, with an incidence rate between 0.5% and 14%, which may cause meningitis or tension pneumocephalus, increasing the risk of reoperation if no intervention is involved in time [8].

Studying the effect of preoperative and intraoperative factors on the occurrence of postoperative CSF Leak can help to foresee the occurrence and development of CSF Leak after transsphenoidal surgery in advance and carry out prevention or treatment in time. In the meta-analysis by Zhou et al. [9], 34 observational studies and 9144 patients were included; gender, age and body mass index, tumor size and scope, tumor texture, and experience level of surgeons were summarized as the main factors of postoperative CSF Leak. However, most of the included studies were Chinese articles, with great implementation bias. In our study, 13 literatures with study sites in different regions around the world were included to quantitatively analyze the possible influencing factors and provide the basis for taking targeted preventive measures.

## 2. Materials and Methods

### 2.1. Search Strategy

The databases Embrase, Medline, PubMed, and Cochrane library were selected as English literature sources for this study, and CNKI and CBM were used as Chinese literature sources. The search was completed in December 2021. Search method: quick search of keywords; combination of keywords: [*Predictors/factors*] AND [*cerebrospinal fluid leak/CSF/Cerebrospinal fluid rhinorrhea*] AND [*pituitary adenoma*] AND [*endoscopic transnasal pituitary surgery/transsphenoidal surgery*].

### 2.2. Inclusion Criteria

(1) All literatures were retrospective observational study papers, which were limited to cohort study or case-control study. There is no limit to the number of research centers. The randomized controlled study, case analysis, noncontinuous time series study, cross-sectional study, and case report study were excluded. (2) The patient was diagnosed with pituitary adenoma by transsphenoidal surgery. After the opening of nasal sphenoid sinus, the incision was made to expose the tumor and scrape off the tumor tissue. (3) CSF Leak: postoperative CSF Leak is defined as the outflow of clear fluid from the saddle or parasellar region within 1-7 days after surgery. Literatures in which the study purpose is intraoperative (non-postoperative) CSF Leak are excluded. (4) Literature review: the patients were divided into 2 groups for factor analysis: the group with postoperative CSF Leak and the group without postoperative CSF Leak, and complete data could be obtained.

### 2.3. Selection of Literatures

Two researchers independently completed the screening of literatures. After the literatures were searched by keywords, the title and abstract of the literatures were read to exclude the literatures that did not meet the requirements, and then, the full text of the literatures was obtained and read to further determine whether they were included. After this, 2 researchers performed a cross-check, and if there is a disagreement between two researchers, a third researcher is invited to step in to resolve it.

### 2.4. Data Extraction

After the included literatures were determined, two institutes further read the literatures; independently extracted the basic information, study characteristics, and outcome indicators of the literatures; and recorded them using excel table. If the data cannot be determined due to incomplete data, the original author should be contacted to obtain all the data; if the data can still not be obtained, the literature will be excluded. In order to facilitate the final statistical analysis, the data expressed as “%” will be converted to the actual number of cases. After completing this work, two researchers cross-checked the extracted data to resolve disagreements and determine the content of the data.

### 2.5. Outcome Indicators

The factors that may cause postoperative CSF Leak in the literatures were collected (in some literatures, it has become *Predictors*), such as gender, age, BMI, tumor size, total resection or hemisection, intraoperative CSF Leak, operation time, cerebral edema, second operation, and preoperative chemotherapy. The information (number of cases and continuous value) of patients with this factor in different groups was obtained.

### 2.6. Literature Quality Evaluation

The Newcastle-Ottawa scale (NOS scale) [7] was used to analyze the quality of the included articles, and the scale was used to evaluate the object selection, comparability, and outcome indicators of the articles. The maximum score was 9 points, and the score of more than 5 points was considered as good quality. The higher the score, the better the literature quality and the less the bias. The Newcastle-Ottawa scale (NOS) is suitable for evaluating case-control studies and cohort studies. It evaluates cohort and case-control studies by means of three large blocks of eight entries, specifically including study population selection, comparability, exposure, or outcome assessment. The NOS evaluation of the quality of the literature employs the semiquantitative principle of star system with a total of 9 stars. NOS has its own dedicated website (http://www.ohri.ca/programs/clinical_epidemiology/oxford.asp). You can see the site if you are interested.

### 2.7. Statistical Analysis

(1) The analysis tool used is the Revman 5.4 software. (2) Use mean difference (MD) to report continuous variables (BMI and tumor size) and odd rate (OR) value and 95% CI to report binary variables (age, whether there is a second operation, whether there is intraoperative CSF Leak), and use forest plot to present the results. (3) *Q* test was used to verify literature heterogeneity. *P* > 0.05 indicated no heterogeneity and good consistency. Fixed effects model analysis could be used to calculate OR the with Mantel-Haenszel method. If heterogeneity existed, random effects model analysis was used to calculate OR with the DerSimonian and Laird method. If fixed effects analysis was consistent with random effects analysis, sensitivity analysis result was stable. (4) Heterogeneity was investigated by subgroup analysis. (5) Funnel plot was used to show the results of publication bias analysis.

## 3. Results

### 3.1. Literature Search

In this study, 584 relevant literatures were initially detected, 211 literatures were filtered out through repeated detection, and the remaining 373 literatures were included in the primary screening, and 13 literatures were finally included. The screening process is shown in Figure 1.

### 3.2. Basic Information of the Included Literatures

13 literatures were included in this study. The basic data, factors, and quality score of the literatures are shown in Table 1.

### 3.3. Excluded Literatures and Reasons for Exclusion

We present 6 excluded articles (not all) after reading the full text, which were excluded mainly because of the following: (a) the study was for intraoperative CSF leakage, (b) no factor analysis, (c) no data available, and (d) patients with nonpituitary tumors, as shown in Table 2.

### 3.4. Meta-Analysis Results

#### 3.4.1. Age

Four literatures [10–13] reported the effect of age on whether patients had postoperative CSF Leak, including 653 patients aged <40 years and 1165 patients aged >40 years. There was no heterogeneity between the literatures (*I*^2^ = 46%, *P* = 0.14). Fixed effects model analysis showed that there was no significant difference in the proportion of patients with CSF Leak in different age groups (OR = 0.71, 95% CI (0.41, 1.20), *P* = 0.20), as shown in Figure 2.

#### 3.4.2. BMI

Seven literatures [14–20] reported the comparison of BMI between patients with postoperative CSF leakage and patients without CSF leakage. There was no statistical heterogeneity between the literatures (*I*^2^ = 0%, *P* = 0.88). Fixed effects model analysis showed that the BMI of patients with postoperative CSF leakage was significantly higher than that of patients without CSF leakage (MD = 2.26, 95% CI (1.31, 3.20), *P* < 0.00001), as shown in Figure 3.

#### 3.4.3. Tumor Size

Four literatures [15, 19–21] reported the comparison of tumor size between patients with postoperative CSF Leak and patients without CSF Leak, with statistical heterogeneity between the literatures (*I*^2^ = 84%, *P* = 0.0003). Random effects model analysis showed that there was significant difference in tumor size between patients with postoperative CSF Leak and patients without CSF Leak (MD = 1.35, 95% CI (0.22, 2.49), *P* = 0.02), as shown in Figure 4.

#### 3.4.4. Whether There Is Second Operation

Four literatures [13, 19, 21, 22] reported whether the type of surgery was secondary surgery affecting the occurrence of postoperative CSF Leak, without statistical heterogeneity between the literatures (*I*^2^ = 37%, *P* = 0.19). Fixed effects model analysis showed that the possibility of CSF Leak in the secondary surgery was higher (OR = 2.20, 95% CI (1.45, 3.33), *P* = 0.0002), as shown in Figure 5.

#### 3.4.5. Intraoperative CSF Leak

Six literatures [12, 13, 18, 19, 21, 22] reported whether intraoperative CSF Leak affected the occurrence of postoperative CSF Leak, with statistical heterogeneity between literatures (*I*^2^ = 81%, *P* < 0.0001). Random effects model analysis showed that the patients with intraoperative CSF Leak were more likely to have postoperative CSF Leak (OR = 8.88, 95% CI (3.64, 21.69), *P* < 0.00001), as shown in Figure 6.

#### 3.4.6. Heterogeneity Investigation and Sensitivity Analysis

In the analysis of tumor size, after the literatures were divided into 2 subgroups according to the calculation method of tumor size, there was no internal heterogeneity, which indicated that the calculation method of tumor size was the source of heterogeneity in the analysis of this factor. The results from the fixed effects model were the same as those from the random effects model in the remaining analyses, indicating that the results were stable.

#### 3.4.7. Analysis of Publication Bias

Publication bias analysis was not performed because few articles were included in the study (Figure 7).

## 4. Discussion

Endoscopic transsellar approach and craniotomy are the two main surgical resection methods for pituitary adenoma. The former is significantly less invasive than the latter, which is a reliable and minimally invasive surgery, but it may still produce complications including cerebrospinal fluid rhinorrhea, epistaxis, olfactory dysfunction, and sinusitis; cerebrospinal fluid leakage is one of the serious complications, which can increase the risk of postoperative intracranial infection (commonly used anti-infective drugs include amoxicillin and metronidazole [23, 24]). The possible cause of CSF Leak is rupture of the top saddle diaphragm or arachnoid membrane caused by resection of the tumor, causing cerebrospinal fluid outflow from the nasal cavity [25]. At present, according to known reports, the incidence of postoperative CSF Leak after endoscopic treatment of pituitary adenoma is between 0.5% and 14% [25, 26]. In this study, the incidence of postoperative CSF Leak was 6.79%, close to 5.6% reported in the literature [9, 26].

The occurrence of CSF Leak may be related to patient's own characteristic factors, tumor characteristic factors, and surgical factors. The reports in various studies are not exactly the same. Therefore, in this meta-analysis, the CSF Leak caused by different factors was summarized and analyzed.

### 4.1. Patient's Own Characteristic Factors

The common factors affecting postoperative CSF leakage include age factor and body mass index (BMI) factor. In the 13 included literatures, gender was not the relevant factor of postoperative CSF Leak. Therefore, no summary analysis is conducted in this study. In this meta-analysis, there was no significant difference in the incidence of postoperative CSF Leak at different age levels, suggesting that age is not a relevant factor for the occurrence of postoperative CSF Leak. However, patients with a postoperative CSF Leak had a significantly higher BMI than those without, suggesting that patients with a higher body mass index (obesity) are more likely to have a postoperative CSF leak, consistent with the observations of some scholars [27, 28]. The pathophysiology of obesity leading to an increased incidence of CSF Leak is uncertain, but the possibility of intracranial hypertension in obese patients was higher; during surgery, persistent elevated intracranial pressure eventually leads to postoperative saddle reconstruction dehiscence, resulting in the occurrence of CSF Leak [27, 29]. Therefore, when time permits, for young and obese patients, preoperative weight loss should be performed, while the operation should more carefully examine whether the intracranial pressure is increased and whether there is intraoperative CSF Leak. Once intraoperative CSF Leak and severe collapse of sellar septum occur, saddle floor reconstruction should be actively performed, and lumbar drainage should be performed when necessary to reduce the intracranial pressure.

### 4.2. Tumor Factors

Many studies [15, 20] have shown that patients with giant adenoma are more prone to have postoperative CSF Leak than microadenoma. This summary shows that patients with CSF Leak have larger tumors (in diameter or volume) than patients without CSF Leak; that means tumor size is one of the factors for the occurrence of CSF Leak. The reason for this is that larger tumors grow parasellar or suprasellar and are more likely to cause injury when surgically removing tumor tissue protruding into the saddle and parasellar region, and the voids left after resection of giant adenomas make the arachnoid membrane on the saddle more likely to collapse and cause damage [30–32]. At the same time, larger tumors as well as tumors with wider invasion to the surrounding can often only be partially resected, while many surgeons pursue near total resection and have a higher risk of CSF Leak and bleeding. Therefore, for larger adenomas, particular attention should be paid to the occurrence of CSF Leak and timely drainage.

### 4.3. Surgical Factors

Our study also found that the incidence of postoperative CSF Leak in patients undergoing reoperation was higher than that in patients undergoing the first operation (OR = 2.20, 95% CI (1.45, 3.33)), which may be due to the formation of scar and tissue adhesion during the first operation, postoperative vascular proliferation, and tissue fibrosis, making it difficult to find the residual part of the tumor during reoperation, increasing the risk of CSF Leak by more invasive anatomical procedures during resection [31–33]. Our study also found that patients with intraoperative CSF Leak had an increased risk of secondary postoperative CSF Leak, which was a risk factor for postoperative CSF Leak, which may be related to insufficient repair of intraoperative cerebral spinal fluid leakage or postoperative buttress changes that caused the leakage to not close due to detachment and displacement of the repair material, or pulsatile cerebrospinal fluid impact on the weak sellar septum, or the subsided sellar septum was punctured by the saddle floor bone margin [23]. Therefore, we believe that skull base reconstruction should be actively performed when cerebrospinal fluid leakage occurs during surgery, and prophylactic lumbar drainage of cerebrospinal fluid should be performed if necessary.

Some literatures reported that the type of tumor, texture of tumor, operation time, and preoperative cerebral edema were also risk factors of postoperative CSF Leak. However, there were few reported literatures, so we could not conduct a summary analysis. Although we found in this meta-analysis that age was not a risk factor for CSF Leak, it remains to be further determined because too few articles were included. In our study results, it was determined that BMI, tumor size, reoperation, and occurrence of intraoperative CSF Leak were related factors of postoperative CSF Leak, which were different from 4 related factors of tumor size, adenoma consistency, reoperation, and intraoperative CSF Leak obtained in the meta-analysis [9], which may be related to different literatures included in the two meta-analyses.

In the analysis of tumor size, we observed significant heterogeneity among the literatures (*I*^2^ = 84%, *P* = 0.0003), but when we divided the 4 literatures into two subgroups according to different methods of tumor size assessment, the internal heterogeneity disappeared (*P* < 50%), indicating that the method of assessment was the source of heterogeneity. We also did not find serious publication bias in the publication bias analysis, but there were still few included literatures based on each risk factor, the coverage of risk factors was not comprehensive enough, and the risk factors for the occurrence of CSF Leak after transsphenoidal surgery for pituitary adenoma are still worthy of continued in-depth discussion.

## 5. Summary

This study included 13 studies on the factors that influence CSF Leak after pituitary adenoma transsphenoidal surgery. According to the findings, BMI, tumor size, reoperation, and the presence of intraoperative CSF Leak were the risk factors for postoperative CSF leak. However, there are still few included literatures based on each risk factor, and the coverage of the risk factors is insufficient, and it is still worthwhile to continue to deeply investigate the risk factors for the occurrence of CSF Leak after pituitary adenoma transsphenoidal surgery.

## Figures and Tables

**Figure 1:** Search and selection chart.

**Figure 2:** Effect of age on CSF Leak after transsphenoidal surgery for pituitary adenoma.

**Figure 3:** Effect of BMI on CSF Leak after transsphenoidal surgery for pituitary adenoma.

**Figure 4:** Effect of tumor size on CSF Leak after transsphenoidal surgery for pituitary adenoma.

**Figure 5:** Effect of secondary operation on CSF Leak after transsphenoidal surgery for pituitary adenoma.

**Figure 6:** Effect of CSF Leak during surgery on CSF Leak after transsphenoidal surgery for pituitary adenoma.

**Figure 7:** Publication bias analysis of the effect of patient BMI on CSF Leak after transsphenoidal surgery for pituitary adenoma.

**Table 1:** Summary of the basic information and risk factors of the included literatures.

Serial number	Author	Study location	Date of publication	Total cases	Number of cases of postoperative CSF Leak (%)	Factors	Quality score (points)
1	Ivan et al. [10]	California, USA	2015	98	11 (11.2)	(a)	6
2	Fraser et al. [14]	Pennsylvania, USA	2018	615	103 (16.7)	(b) and (c)	6
3	Patel et al. [15]	Vanderbilt, USA	2018	806	38 (4.7)	(b), (c), and (d)	5
4	Zhang et al. [11]	Shanghai, China	2017	474	13 (2.7)	(a) and (e)	5
5	Karnezis et al. [16]	Multicenters of Australia, Canada, and USA	2016	1161	68 (5.9)	(b), (d), and (h)	7
6	Q. Liu et al. [12]	Xuzhou, China	2020	194	25 (12.9)	(a), (d), and (f)	5
7	Tian et al. [13]	Yantai, China	2018	1063	29 (2.7)	(a), (d), (e), (f), and (h)	5
8	Sun et al. [17]	Singapore	2018	123	10 (8.1)	(b)	6
9	Liu et al. [22]	Guangdong, China	2012	397	31 (7.8)	(e) and (f)	5
10	Hannan et al. [18]	Austria	2020	270	24 (9)	(b) and (f)	5
11	Dlouhy et al. [19]	Iowa, USA	2012	96	13 (13.5)	(b), (d), (e), and (f)	6
12	Lee et al. [20]	Los Angeles, USA	2020	78	14 (17.9)	(b), (d), (g), and (h)	6
13	Han et al. [21]	Guangzhou, China	2008	592	26 (4.4)	(b), (e), and (f)	6

Notes: (a) age; (b) BMI; (c) hydrocephalus; (d) tumor size; (e) secondary surgery; (f) intraoperative CSF leaks; (g) operation time; (h) radiation therapy before surgery.

**Table 2:** Excluded literatures and reasons for exclusion (not all).

Serial number	Author	Date of publication	Reason for exclusion
1	Zhou et al. [34]	2017	Not postoperative CFL (intraoperative)
2	Lee et al. [35]	2019	No risk factors of CFL
3	Campero et al. [36]	2019	Not postoperative CFL (intraoperative)
4	Xue et al. [37]	2020	No data available
5	Nishioka et al. [38]	2005	Not pituitary adenomas patients
6	Cheng et al. [23]	2018	Not postoperative CFL (intraoperative)

## Data Availability

The simulation experiment data used to support the findings of this study are available from the corresponding author upon request.
